# MicroRNA-155-5p modulates the progression of acute respiratory distress syndrome by targeting interleukin receptors

**DOI:** 10.1080/21655979.2022.2071020

**Published:** 2022-05-04

**Authors:** Zhenfei Huang, Hui Huang, Meirong Shen, Changrong Li, Chao Liu, Huayong Zhu, Weiwei Zhang

**Affiliations:** a Department of ICU, GanZhou People`s Hospital, Ganzhou, Jiangxi, China; b Department of medical, GanZhou People`s hospital, Ganzhou, Jiangxi, China

**Keywords:** MicroRNA-155-5p, acute respiratory distress syndrome, interleukin receptor, NF-kB pathway

## Abstract

Acute respiratory distress syndrome (ARDS) is a multifactorial inflammatory lung failure with a high incidence and a high cost burden. However, the underlying pathogenesis of ARDS is still unclear. Recently, microRNA has been shown to have critical function in regulating the pathogenesis of ARDS development and inflammation. To identify the important microRNA in the serum from patients with ARDS that may be potential biomarkers for the disease and explore the underlying disease mechanism. We found significant upregulation of miR-155-5p expression in serum samples from patients with ARDS compared with the control group (p < 0.01). The levels of interleukin receptors and inflammatory cytokines were significantly increased in blood samples from patients with ARDS (p < 0.05). In the cell model, miR-155-5p had a binding site in the 3’-UTR of the three interleukin receptors. In LPS-simulated BEAS-2B cells, transfection of miR-155-5p mimic inhibited the expression levels of these interleukin receptors, and was found to directly target the inflammatory response of leukocyte nodulin receptor through NF-kB signaling. In conclusion, miR-155-5p can alleviate LPS-simulated injury that induces the expression of IL17RB, IL18R1, and IL22RA2 by affecting the NF-kB pathway; however, it cannot change the occurrence of inflammatory storms. Collectively, this suggests that the progression of ARDS is the result of effects of the multiple regulatory pathways, providing novel evidence for the therapy of ARDS.

## Highlights

- miR-155-5p alleviate LPS-simulated injury.
- miR-155-5p induces the expression of IL17RB, IL18R1, and IL22RA2.
- miR-155-5p induces the NF-kB pathway.

## Introduction

Acute respiratory distress syndrome (ARDS) is a destructive immune response characterized by inflammation, lung permeability, and edema, which lead to life-threatening acute injury to lung epithelial and endothelial cells [1,2]. The onset of the syndrome is acute, for example 24 to 48 hours or 5 to 7 days. The clinical manifestations included acute respiratory failure, obvious hypoxia, and bilateral invasion on chest imaging, accompanied by chest tightness, cough, and blood phlegm [3,4]. Various clinical diseases are closely related to the progression of ARDS; the rates of incidence and mortality are significant, contributing significantly to the hundred thousand patients admitted to intensive care units (ICUs) each year. The pathogenesis of ARDS is complex, with various causes; common causes include sepsis, pneumonia, and aspiration, but there are also less common risk factors [2,5,6]. Therefore, its differential diagnosis is more difficult and mainly dependent on imaging and other clinical manifestations. At present, ARDS represents a huge social burden, seriously affects patients’ quality of life, and causes increased costs and usage of healthcare services [7–9]. Limited by unsuccessful targeted treatments, the treatment of ARDS has consisted of mainly supportive care. The mechanism of ARDS is still unclear.

MicroRNAs (miRNAs) are noncoding RNAs composed of 20–23 nucleotide double bonds that can interact with specific targets on messenger RNAs (mRNAs) to regulate gene expression, thereby functioning as inhibition or degradation targets. In general, their expression levels change dynamically in different states of the body, and participate in various cell processes, including viability, differentiation, apoptosis, the immune response, and different pathological processes [10–12]. Therefore, the real-time detection of miRNAs can reveal the pathological changes in related cells or tissues and provide functional information on disease development [13]. In particular, miRNAs are relatively well conserved throughout evolution and relatively stable in blood samples, demonstrate their sensitivity as prognostic biomarkers. Transcriptome data have confirmed the involvement of microRNAs in various human diseases, including ARDS, sepsis, liver cancer, and lung cancer [14–17]. It has been shown that miR-155-5p expression in the serum of patients with ARDS is significantly higher than that of the control, indicating that this miRNA is closely associated with the progression of ARDS and is an important factor in ARDS. However, the gene targets of miR-155-5p are unclear.

In the current study, we found that miR-155-5p was highly expressed in patients with ARDS and LPS-stimulated BEAS-2B cells. In addition, three potential targets of miR-155-5p, interleukin 17 receptor B (IL17RB), interleukin 18 receptor 1 (IL18R1) and interleukin 22 receptor subunit alpha 2 (IL22RA2), have been investigated, indicating it is a modulator of ARDS progression. However, the inflammatory cytokine infiltration and pathological progression could still not be alleviated. These results provide a novel mechanism by which the inflammatory response is regulated in multiple pathways and should be investigated in further studies.

## Methods

### Clinical samples

Thirty patients with ARDS and thirty healthy volunteers were enrolled in the research. The study was approved by the Medical Ethics Committee of GanZhou People’s hospital. All participants were given details of the study and signed informed consent.

### Cell culture and treatment

The BEAS-2B, A549 cell line, which is a human alveolar epithelial cell line, was acquired from the American Type Culture Collection (ATCC). BEAS-2B, A549 cells were cultivated in DMEM containing with 10% FBS (Invitrogen, China) in a 37°C incubator. When the cells reached 70%–80% confluence, they were seeded into 24-well plates for further experiment. Lipopolysaccharide (LPS; Sigma-Aldrich, Shanghai, China) was prepared at 5 mg/mL in PBS buffer, and then added into cultured cells at a final concentration of 10 µg/mL to establish the ARDS model [14–17]. Subsequently, miR-155-5p mimic (50 nM) or miR-155-5p inhibitor (50 nM) was transiently transfected into the cells using Lipofectamine 2000 (Invitrogen, China). After transfection, the cells were used for further experiments.

### qRT-PCR assay

The treated cells were harvested and incubated with TRIzol reagent (Invitrogen, China). Total RNA was extracted from these cells and 1.0 µg of RNA was directly utilized for reverse transcription into cDNA by PrimerScript RT Master Mix kit (Takara, Dalian, China) following the manufacturer’s instructions. The resultant cDNA was analyzed by qPCR using SYBR Green Universal Master mix (Roche Diagnostics). All primers utilized in the study were acquired from Sangon Biotech (Shanghai). U6 and GAPDH were utilized as the internal controls to normalize the Ct values for miR-155-5p and the inflammatory cytokine receptors, respectively, to determine their relative expression.

### ELISA analysis

To investigate the release of inflammatory cytokine receptors, the levels of IL17RB, IL18R1, and IL22RA2 in the cell supernatant were measured. In brief, LPS reagent was injected into the medium for 24 hours and the relative levels of human IL17RB (EK0785), IL18R1 (EK1260), IL22RA2, IL-1β, IL-6, IL-8, and TNF-α were measured in the treated cells using an ELISA kit (Boster, Wuhan, China) in accordance with the manufacturer’s protocol [14–17].

### Bioinformatic analysis

To explore the potential target genes of miR-155-5p, TargetScan [18] was applied. Based on the results, three inflammatory cytokine receptors – IL17RB, IL18R1, and IL22RA2 – were selected from all the predicted targets.

### Dual-luciferase reporter system

In brief, the 3’-UTR the three inflammatory cytokine receptors was constructed into a luciferase vector pmirGLO (Promega, Beijing, China) to produce WT IL17RB, IL18R1, and IL22RA2 3’-UTR reporters. A site-directed mutagenesis kit (Takara) was utilized to generate the mutants on the potential interaction sites. Either WT or MUT constructs were co-transfected with either miR-155-5p mimic or miR-NC via Lipofectamine2000. After transfection for 48 hours, the relative luciferase activity has been finally measured.

### Western blotting assay

The treated cells were harvested and incubated with RIPA lysis buffer (BiYunTian, Shanghai) on ice for 1 hour. Subsequently, all samples were centrifuged at 10,000 rpm for 10 minutes. Bradford method was used to determine the protein concentration. Then, 10 µg concentration of protein from each sample was separated by SDS-PAGE and transferred to a polyvinylidene fluoride membrane. Nonspecific binding to the membrane was blocked by incubation in 5% skimmed milk. After three washes with PBS, the membrane was incubated with the selected primary antibody at 4°C overnight. Subsequently, after appropriate washing, the membrane was incubated with secondary antibody for 1 hour. Finally, the protein bands were visualized using a membrane-enhanced chemiluminescence (ECL) reagent kit and the band intensity was quantified by 3.2 AlphaImager 2200 software.

### Statistical analysis

Results from independent experiments conducted in triplicate were examined using SPSS software (SPSS, Chicago) and present as the mean ± standard deviation. Results were compared using Student’s *t*-test or ANOVA. A p value of < 0.05 was considered to indicate a statistically significant difference.

## Results

### Upregulation of miR155-5p in the ARDS model

The expression level of miR-155-5p was detected in samples of serum from patients with ARDS. As shown in Figure 1(a), there was a significant increase in the expression of miR-155-5p in patients with ARDS. A similar result was found for miR-155-5p expression in the cell model of ARDS (LPS-stimulated BEAS-2B cells), which showed an increase compared with control cells (Figure 1(b)). These results imply that miR-155-5p may be associated with the progression of ARDS, which is consistent with the previous study [14–17].

**Figure 1.** Upregulated expression of miR-155-5p in ARDS and LPS-stimulated BEAS-2B cells. The expression levels of miR-155-5p in serum samples from patients with ARDS (a) and in LPS-stimulated BEAS-2B cells (b). **p < 0.01 compared with the control.

### MiR-155-5p directly targeted IL17RB, IL18R1, and IL22RA2

To investigate the mechanism through which miR-155-5p affects ARDS, the possible targets were predicted by bioinformatic methods and confirmed using a dual-luciferase reporter system. After bioinformatic screening, we identified that IL17RB, IL18R1, and IL22RA2 had potential binding sites for miR-155-5p in the 3ʹUTR (Figure 2(a)). As expected, miR-155-5p mimic significantly inhibited luciferase activity when transfected with the WT, but not with MUT (Figure 2(b)). The targeting of IL17RB, IL18R1, and IL22RA2 by miR-155-5p was then determined in LPS-stimulated cells. The results showed that the relative levels of IL17RB, IL18R1, and IL22RA2 were significantly decreased in BEAS-2B cells transfected with miR-155-5p mimic compared with the control group. In addition, the levels of IL17RB, IL18R1, and IL22RA2 were significantly increased in BEAS-2B cells transfected miR-155-5p inhibitor than the control group (Figure 2(c)).

**Figure 2.** Identification of IL17RB, IL18R1, and IL22RA2 as potential targets of miR-155-5p. IL17RB, IL18R1, and IL22RA2 were identified as potential targets of miR-155-5p by the databases (a); this was confirmed by the dual-luciferase report assay (b). The levels of IL17RB, IL18R1, and IL22RA2 were measured by qRT-PCR (c). *p < 0.05 and **p < 0.01, ANOVA.

### Clinical characteristics

There were 30 cases of ARDS, with an average age of 20. Among them, there were 17 males, 13 females, average pH = 7.20 + 0.25, PaCO_2_ = 3.5 + 1.21, PaO2 = 8.63 + 3.2. The basic diseases included 13 respiratory diseases, and the rest were nervous system and hepatitis. As a control, 30 healthy people were selected with average age of 20, and there were 15 males and 15 females.

### Upregulation of inflammatory factors in patients with ARDS

To explore the expression of inflammatory cytokine receptors in patients of ARDS, the mRNA levels of IL17RB, IL18R1, and IL22RA2 were measured by qRT-PCR. As shown in Figure 3(a), the expression of these receptors was significantly increased in patients with ARDS compared with healthy volunteers. Next, the serum concentrations of these factors were detected by ELISA. There was a significant increase in the levels of inflammatory cytokine receptors (Figure 3(b)) and the important inflammatory cytokines (Figure 3(c)). Notably, the cytokine storm is an important regulator of the progression of ARDS.

**Figure 3.** Upregulated levels of the inflammatory cytokines in patients with ARDS. The levels of IL17RB, IL18R1, and IL22RA2 in serum samples from patients with ARDS (a). Serum concentrations of IL17RB, IL18R1, and IL22RA2 (b), and IL-1β, IL-6, IL-8, and TNF-α (c) in patients with ARDS were analyzed by ELISA. *p < 0.05, **p < 0.01, and ***p < 0.001 compared with the control.

### Relative expression of NF-kB following LPS-stimulated injury

We measured the relative expression levels of NF-kB in LPS-stimulated A549. The qRT-PCR analysis indicated that the relative level of NF-kB expression was significantly higher in the LPS-stimulated group than in the control group. The relative mRNA expression levels of NF-kB, STAT1, and STAT3 in LPS-stimulated cells were significantly increased in expression (Figure 4(a)). This change was confirmed at the protein level by western blotting assay (Figure 4(b)). These findings demonstrated that LPS significantly promoted the expression of NF-kB, STAT1, and STAT3 compared with the control group.

**Figure 4.** Relative expression level NF-kB following LPS stimulation. The expression levels of NF-kB were evaluated by qRT-PCR (a) and western blotting (b) in LPS-stimulated human alveolar epithelial cells. *p < 0.05, **p < 0.01, and ***p < 0.001 compared with the control.

### Suppression of NF-kB signaling by miR-155-5p probably occurs through the inflammatory cytokine receptors

To examine the relationship between miR-155-5p and NF-kB signaling, western blotting was performed to measure the relative expression levels of NF-kB. As shown in Figure 5, the expression levels of IL17RB, IL18R1, and IL22RA2 in LPS-stimulated BEAS-2B cells transfected with miR-155-5p mimic were significantly decreased compared with the control group. Most importantly, inhibitory effects on the miR-155-5p mimic on NF-kB signaling were detected. Collectively, these results imply that miR-155-5p modulates NF-kB signaling in LPS-simulated BEAS-2B cells by modulating the level of the inflammatory cytokine receptors.

**Figure 5.** miR-155-5p inhibited the NF-kB signaling pathway. The expression levels of the inflammatory cytokine receptors (IL17RB, IL18R1, and IL22R2) and NF-kB-related proteins (NF-kB, STAT1, and STAT3) were measured by western blotting analysis with β-actin used as the internal control. *p < 0.05, **p < 0.01, and ***p < 0.001 compared with the control.

## Discussion

ARDS is a severe lung inflammatory disease that induces multiple organ failure with a high incidence and mortality rate [19,20]. As the molecular mechanism of ARDS is still unknown, the treatment of ARDS is mainly through supportive therapy. Recent high-throughput screening studies in patients with ARDS and animal models have found that differential expression of miRNAs is widespread during the progression of lung diseases, and exerts critical functions relating to inflammation and apoptosis [21–23]. Microarray analysis showed that the level of miR-802 was significantly downregulated in a mouse model of ARDS. The overexpression of miR-802 could significantly suppress the generation of inflammatory cytokines induced by LPS in vitro, and significantly alleviate LPS-simulated acute lung injury [24]. The expression of miR-150 in the serum of patients with ARDS was significantly decreased and negatively correlated with the severity of ARDS [25]. Clearly, miRNA as a biomarker or target of drug therapy has good application prospects.

In this study, we showed that the level of miR-155-5p was significantly decreased in the serum of patients with ARDS, which was consistent with the previous results [26]. Interestingly, the dual-luciferase activity assay confirmed that the proinflammatory cytokine receptors IL-17 RB, IL-18R1, and IL22RA2 were possible target genes of miR-155-5p; however, the serum content of these factors was increased. Furthermore, the relative expression of IL-6, IL-1β, IL-8, and TNF-α has was significantly increased in patients with ARDS and LPS-induced BEAS-2B cells transfecting with miR-155-5p mimic compared with the control group. Although the expression of IL-17 RB, IL-18R1, and IL22RA2 was downregulated by miR-155-5p, these changes could not promote an anti-inflammatory state. There is growing evidence that the major cause of ARDS is the imbalance between the inflammatory and anti-inflammatory responses, accompanied by increased levels of pro-inflammatory cytokines [2,27,28]. The important inflammatory cytokines (IL-6, IL-1β, IL-8, and TNF-α) participated the initiate cascade inflammatory responses and led to a change in inflammatory cytokine infiltration [29]. The elevated levels of these pro-inflammatory factors contributed to tissue injuries, modulated inflammation, and induced cell apoptosis [30].

Nuclear factor-kappa B (NF-kB) is characterized as a unique nuclear transcription factor and found widely in higher eukaryotes, mainly in the form of a dimer. There is increasing evidence to show that NF-kB signaling is closely associated with the expression of a variety of inflammatory cytokines and that it has a critical function in the progression of ARDS [31,32]. However, the regulatory mechanism of NF-kB is still unclear. Here, we showed that NF-kB-related genes were upregulated in LPS-stimulated A549. However, miR-155-5p could directly target the inflammatory factor receptors IL17R, IL18RB, and IL22R2, suppressing the NF-kB signaling pathway and thus inhibiting the inflammatory responses. This suggests that although miR-155-5p overexpression can suppress NF-kB signaling, it cannot alleviate the inflammatory response in ARDS progression. Together, these findings suggest that the immune response process in ARDS is regulated and coordinated by multiple pathways.

Our study is not without limitations. The interaction between miRNA and its targets is complex. Further research is needed to determine the underlying functions of miR-155-5p in the ARDS model. Furthermore, we characterized the mechanism of miR-155-5p in BEAS-2B cells. This is an adenocarcinomic human alveolar basal epithelial cell line and is therefore not representative of normal bronchial or lung epithelial cells. However, recent studies have used BEAS-2B cells to explore LPS-induced inflammation, which is also an important miR-155-5p-targeted pathway (IL17R, IL18RB, and IL22R2) [18,33–35].

## Conclusion

miR-155-5p expression is upregulated in patients with ARDS and LPS-stimulated A549. In LPS-stimulated ARDS, the NF-kB signaling pathway is induced. However, miR-155-5p directly targets IL17R, IL18RB, and IL22R2, thus suppressing the downstream NF-kB signaling pathway. These results may provide a wider understanding of the progression of ARDS.

## Abbreviations

ARDS: acute respiratory distress syndrome; LPS: lipopolysaccharide; miRNA: microRNA; mRNA: messenger RNA; IL17RB: interleukin 17 receptor B; IL18R1: interleukin 18 receptor 1; IL22RA2: interleukin 22 receptor subunit alpha 2; ATCC: American Type Culture Collection.
